The article "Evaluation of queen cell acceptance and royal jelly production between hygienic and non-hygienic honey bee (Apis mellifera) colonies" was retracted in 2022. Reasons: compromised peer review; a conflict of interest; concerns about the authorship.

# Evaluation of queen cell acceptance and royal jelly production between hygienic and non-hygienic honey bee (*Apis mellifera*) colonies

**DOI:** 10.1371/journal.pone.0266145

**Published:** 2022-03-28

**Authors:** Khalid Ali Khan, Hamed A. Ghramh

**Affiliations:** 1 Research Center for Advanced Materials Science (RCAMS), King Khalid University, Abha, Saudi Arabia; 2 Unit of Bee Research and Honey Production, Faculty of Science, King Khalid University, Abha, Saudi Arabia; 3 Biology Department, Faculty of Science, King Khalid University, Abha, Saudi Arabia; Sivas Bilim ve Teknoloji Universitesi, TURKEY

## Abstract

Honey bees are crucial for pollination services globally and produce important hive products including honey, royal jelly, pollen, and propolis that are being used commercially in food, cosmetics, and alternative medicinal purposes. Among the bee products, royal jelly (RJ) has long attracted scientists’ interest because of its importance in honey caste differentiation. The present research was carried out to determine the acceptance rate of queen cells, and RJ production between the hygienic and non-hygienic lines. Further, this study unveils the effect of pollen substitute diets on the queen cell acceptance rate and RJ yields between both bee stocks. Results showed that the uncapped brood cells and dead brood’s removal percentage was significantly more in hygienic bee colonies in comparison to non-hygienic bee colonies (p < 0.05). The average percentage of larval acceptance was statistically higher in hygienic lines (64.33 ± 2.91%) compared to non-hygienic lines (29.67 ± 1.20%). Similarly, the RJ mean weight per colony differed statistically between both bee stocks (p<0.001), which were 12.23 ± 0.52 g and 6.72 ± 0.33 g, respectively. Moreover, our results demonstrated that a significant difference was observed in larval acceptance rate, RJ yields (per colony and per cup) between both bee stocks those fed on various diets. However, no significant difference was recorded in RJ yields (per colony and per cup) between both bee stock that feeds on either commercially available pollen or pollen substitute. This study may provide future applications in helping bee breeders to choose the bees that carry a higher level of hygienic behavior with high RJ production traits.

## Introduction

Honey bees and other pollinators play a critical role in the ecosystem’s health [1, 2]. Honey bees play a significant role in both agricultural and wild crop pollination due to their ease of transportation, enormous numbers, and level of domestication [3]. Approximately one-third of agricultural crops rely on bees pollinations [4]. The worth of these pollination services is generally calculated in billions of dollars, contributing roughly 9.5 percent to the global value of crops [5, 6]. Additionally, honey bees produce various natural products such as honey, royal jelly, bee bread, propolis, and wax that are used in food, cosmetics and the medicinal industries [7]. However, in the last two decades, dramatic honey bee colonies losses have been recorded in various regions worldwide [8]. It was documented that the honey bee population declined because of several reasons such as destruction of habitat, pesticides, agricultural parasites and pathogens, industrial revolutions, climatic changes, and inadequate food supply [9–12]. Notably, pollen and nectar are the only sources of nutrition for honey bees during their annual colony cycle [13, 14]. In addition, pollen provides proteins, lipids, vitamins and minerals, while supplies primary carbohydrates [15]. Interestingly, first three days of larval growth, both queen and bee worker larvae are fed on the royal jelly (RJ), after, the worker bees larvae fed on combination of RJ and food store (pollen and honey) while queen continues to fed on RJ from worker nurse bees [16]. In addition, honey bee queen rearing is the most important beekeeping practice for rapid multiplication of bee population, as well as replacing old queen every year to enhance honey and RJ production [17].

The article "Evaluation of queen cell acceptance and royal jelly production between hygienic and non-hygienic honey bee (Apis mellifera) colonies" was retracted in 2022. Reasons: compromised peer review; a conflict of interest; concerns about the authorship.

RJ is a yellowish or white pretentious substance which secreted from the various young worker bees’ glands including mandibular, hypopharyngeal, postcerebral, and thoracic glands [18, 19]. It was documented that RJ contributes to the distinct attribute of queens including their fertility, longevity and memory performance [20]. RJ is mainly comprised of water, protein (majority of proteins: major royal jelly protein (MRJPs) and the small number of proteins: royalism, jelleines, and aspimin), lipids, carbohydrates, vitamins and minerals [21]. RJ has shown a wide range of health-promoting effects including antioxidant, antidiabetic, antitumor, antimicrobial, neurotrophic, antirheumatic, and anti-ageing [20, 22]. Recently, RJ has also been documented as a medicinal agent used to ameliorate postmenopausal pathologies [23], Alzheimer’s disease [20]. RJ could be produced for commercial purposes and its demand is increasing every year, and economic value is significantly higher as compared to other honey bee products including honey, pollen, propolis, and venom [24–26]. For example, China is a major producer and seller of RJ, producing approximately 4000 tons per year and accounting for more than 90% of global RJ production. RJ is mostly shipped to the United States, Japan, and European countries [16, 27, 28]. Additionally, some other countries are also the main producer and exporters of RJ including Japan, Korea, Spain, Italy, and France [16, 29].

The article "Evaluation of queen cell acceptance and royal jelly production between hygienic and non-hygienic honey bee (Apis mellifera) colonies" was retracted in 2022. Reasons: compromised peer review; a conflict of interest; concerns about the authorship.

The amount and quality of RJ production are affected by a variety of biotic and abiotic variables [30]. The most important among them are; honey bee races [28, 31], whether the colony is queenless or queenright [32], larval age [33], types of queen cell cups [34], grafting methods [35], queen cell position on grafting bar [36, 37], harvesting time [38], nutritional source [21, 39, 40], season and, also colony strength [37, 41]. When bees feed sugar syrup, for example, the quantity and structure of essential RJ ingredients including amino acids, carbohydrates, and vitamins are significantly altered [42]. Although beekeepers are quite well in and equipped with this manufacturing method, technological improvements can help boost RJ production. To boost RJ output, apicultural scientists are putting in a lot of work to develop new equipment, grafting processes, and selecting high-producing honey bee types.

The current study was carried out to compare the uncapping and removal percentage between hygienic and non-hygienic colonies. Further, to determine the larval acceptance rate and RJ yields difference between hygienic and non-hygienic colonies. In addition, to unveil the effect of different pollen substitutes on RJ yield of both bee stocks. This study may be useful for the breeder in selecting better bee colonies that indicate a higher level of hygienic behavior and produce high RJ in the optimized honey bee’s population.

## Materials and methods

### Measuring of hygienic behavior by the freeze-killed method

Two different populations of *Apis mellifera* were compared regarding their hygienic behavior. The experiment was conducted in 10 honey bee colonies with a one-year-old queen. All full-sized bee colonies had fertile queens, workers, capped and uncapped broods, excessive amounts of food store, and were kept in standard Langstroth hives. The degree of hygienic behavior was measured by minor modification in the method described by Spivak and Gilliam [43]. Briefly, a pin-killed brood assay was performed, 100 cells of capped brood were selected and the brood larvae were killed, and then the brood frame was returned into their respective hives. The percentages of uncapped and dead brood removal in each colony were recorded after 12, 24, and 48 h.

### Measuring of acceptance rate of queen cells

Five colonies of each bee stock were selected for the experiment to investigate the larval acceptance rate between hygienic and non-hygienic colonies. Two hour before the grafting, the grafting frame was inserted in the rearing colonies for polishing and worker larvae (less than one day) were grafted in one frame containing 126 plastic queen cell cups, then introduced to both hygienic or non-hygienic colonies. The frame was removed from the colony after 3 days to examine larval acceptance and RJ yield, as per usual procedure [44, 45]. This study was conducted three times with three-day gaps between each occasion.

The article "Evaluation of queen cell acceptance and royal jelly production between hygienic and non-hygienic honey bee (Apis mellifera) colonies" was retracted in 2022. Reasons: compromised peer review; a conflict of interest; concerns about the authorship.

### Measuring of RJ yield

As followed the above experiment, the wax on the plastic cells’ tops and the larvae inside the cells were taken out. Microspatula was used to collect RJ from the cells into a plastic container, and its weight was calculated with an electronic scale (AL204-IC, Mettler Toledo, Switzerland). RJ was collected and stored at -20°C in the fridge.

### The impact of different nutritional diets on RJ yield

To investigate the nutritional effect on larval acceptance and RJ yields, honey bee colonies were divided into three groups. Commercially available pollen was purchased from the local market and supplied to the first group (hygienic) as a dough. Whereas pollen substitutes (soybean flour + brewer’s yeast powder) were fed to the second group (non-hygienic). In control group, only sugar syrup (50% sucrose w/v) was supplied.

### Statistical analysis

The data about killed brood removal, larval acceptance and RJ yields were measured and analyzed using SPSS software (version 26). The significant difference between two group was determined by Student’s t-test and more than two by Tukey post-hoc test. The data were compared at the 0.05 level.

## Results

### Uncapping and removal percentage of dead brood

The uncapping and removal percentage of dead brood was recorded between hygienic and non-hygienic bee colonies (**Fig 1A and 1B**). Overall, the uncapping percentage of broods differed significantly between hygienic and non-hygienic beelines over a period of time (F (2, 84) = 6.570, p = 0.002). After 24 h, the uncapping percentage of brood cells was 44.00 ± 3.59% in hygienic lines and 10.47 ± 3.32 in non-hygienic bee colonies. The uncapping percentage of dead brood was 68.00 ± 4.05% and 15.13 ± 3.74% after 24 h in both bee stocks, respectively. After 36 h, the uncapping percentage of hygienic lines was 83.27 ± 4.47, which was significantly different from the non-hygienic lines, which was 22.33 ± 4.03%.

**Fig 1:** The uncapping and removal percentage of dead brood between hygienic and non-hygienic bee line over time of inspection. (a) the uncapping percentage of brood cells between both bee stocks after, 12, 24, and 36 h, respectively. (b) the removal percentage of dead broods between both bee stocks after, 12, 24, and 36 h, respectively.

The article "Evaluation of queen cell acceptance and royal jelly production between hygienic and non-hygienic honey bee (Apis mellifera) colonies" was retracted in 2022. Reasons: compromised peer review; a conflict of interest; concerns about the authorship.

Similarly, the result indicated (**Fig 1B**) that dead broods removal percentage was statistically different between hygienic and non-hygienic bee colonies at the inspection (F (2, 84) = 9.391, p = 0.001). It was noticed that the dead broad removal percentage differed significantly between hygienic and non-hygienic colonies after 12 h, that was 39.73 ± 4.16% and 7.73 ± 2.54%, respectively. After 24 h, the removal percentage of dead brood was 62.67 ± 4.78% and 11.60 ± 2.93% between both bee stocks, respectively. After 36 h, the maximum removal percentage of dead broods was 81.53 ± 4.51 in hygienic lines while 16.87 ± 3.19% in non-hygienic lines.

### Larval acceptance rate

The difference in larval acceptance rates between the hygienic and non-hygienic colonies are described (**Fig 2**). The findings showed that larval acceptance rate was statistically more in hygienic colonies than non-hygienic lines (t = 21.977, p = 0.001). On the other hand, no significant difference was recorded in the larval cell acceptance rate within both bee stocks. The highest rate was 64.33 ± 2.91% in the case of hygienic colonies, while 29.67 ± 1.20% in non-hygienic bee colonies.

**Fig 2:** The mean larval acceptance rate of hygienic and non-hygienic bees from ten colonies (five each) over three collection time points.

### Royal jelly yields

The average weight of RJ per colony (g) and per cup (mg) between hygienic and non-hygienic beelines is mentioned, respectively (**Fig 3A and 3B**). The RJ yield was statistically greater in hygienic bee stock in comparison to non-hygienic bee colonies (t = 9.005, p< 0.001). The maximum RJ yield was 12.23 ± 0.52 g in hygienic bee colonies, while in the case of non-hygienic colonies was 6.72 ± 0.33 g.

**Fig 3:** The mean weight (shows as mean ± SE) of Royal Jelly (RJ) collection between hygienic and non-hygienic around 72 h after larval grafting. (a) RJ yield in grams/ colony after 72 h harvesting. (b) RJ yield mg/ cell cup between both bee colonies.

Similarly, the RJ yield per cell cup was statistically more in hygienic bee stock as compared to non-hygienic bee colonies (t = 22.662, p< 0.001). In hygienic bee stocks, the highest RJ yield was 234. 99 ± 2.22 mg, whereas 158.87 ± 2.52 mg/ cell cup in non-hygienic bee colonies. Regarding RJ yield per colony and per cell cup, no significant difference was observed within both honey bee stocks.

### The effect of various nutritional diets on royal jelly yield

Nutritional effect on larval acceptance and RJ yield is mentioned (see **Table 1**). Larval acceptance rate differed statistically inside hygienic bee stocks by feeding different diets including commercially available pollen, pollen substitute, and sugar solution (F (2,15) = 110.368, P< 0.001). Larval acceptance rate differed statistically within the non-hygienic bee stocks (F (2,15) = 13.568, P< 0.001).

The article "Evaluation of queen cell acceptance and royal jelly production between hygienic and non-hygienic honey bee (Apis mellifera) colonies" was retracted in 2022. Reasons: compromised peer review; a conflict of interest; concerns about the authorship.

**Table 1:** The effect of nutritional diets on the queen cell acceptance rate, royal jelly/ colony/cell cup between hygienic and non-hygienic bee colonies.

Diet	Hygienic bee colonies			Non-Hygienic bee colonies		
	Queen cell acceptance rate (%) (Mean ± SE)	Weight (g) of RJ/ colony (Mean ± SE)	Weight (mg) of RJ/ cell cup (Mean ± SE)	Queen cell acceptance rate (%) (Mean ± SE)	Weight (g) of RJ/ colony (Mean ± SE)	Weight (mg) of RJ/ cell cup (Mean ± SE)
Commercially available pollen	65.67 ± 1.45% a	13.62 ± 0.6 a	239.62 ± 2.74 a	32.17 ± 1.89% a	6.63 ± 0.52 a	160.39 ± 4.36 a
Pollen substitute	57.67 ± 1.64% b	12.17 ± 0.74 a	235.89 ± 3.55 a	28.33 ± 1.05% a	5.68 ± 0.28 a	153.45 ± 3.16 a
Sugar syrup	36.83 ± 1.08% c	8.63 ± 0.51 b	221.48 ± 2.55 b	21.83 ± 1.67% b	4.73 ± 0.13 b	141.54 ± 2.17 b

Results are means ± standard errors of triplicate determinations. Means in a column with different letters are significantly different (P< 0.05).

But no significant difference was observed in non-hygienic beelines fed either on pollen or pollen substitute (**Fig 4A**). Regarding commercially available pollen, the larval acceptance rate was greater in the hygienic bee stocks compared to non-hygienic bee stocks (t = 14.066, p< 0.001), which was 65.67 ± 1.45% and 32.17 ± 1.89%, respectively (**Fig 4B**).

**Fig 4:** The nutritional effect on the larval acceptance (shows as mean ± SE) between hygienic and non-hygienic colonies. (a) The overall effect of diet on queen cell acceptance rate between both bee stocks, (b) The effect of pollen diet on queen cell acceptance rate between both bee stocks (c) The effect of pollen substitute diet on queen cell acceptance rate between both bee stocks (d) The effect of sugar syrup on queen cell acceptance rate between both beelines.

In pollen substitute groups, the larval acceptance rate differed significantly between hygienic and non-hygienic bee colonies (t = 14.780, p = 0.001). The larval acceptance rate was 57.67 ± 1.64% in hygienic bee colonies, whereas in hygienic bee colonies was 28.33 ± 1.05% (**Fig 4C**). Similarly, the larval acceptance rate differed statistically between both beelines those fed on sugar solution (t = 9.445, p< 0.001) (**Fig 4D**). The larval acceptance rate was 36.83 ± 1.08% and 21.83 ± 1.67% in both bee stocks.

Nutritional effect on RJ production was investigated between both bee stocks (**Fig 5A**). The RJ yield differed statistically between hygienic bee stocks by feeding on various diets such as commercially available pollen, pollen substitute, and sugar solution (F (2, 15) = 16.949, P< 0.001). In hygienic bee stocks, the RJ yield was 13.62 ± 0.6 g, 12.17 ± 0.74 g, and 8.63 ± 0.51g in the case of pollen diet, pollen substitute, sugar syrup, respectively (**Fig 5A**). In non-hygienic bees, no significant difference was found in the mean weight of RJ yield those bee colonies either fed on pollen (6.63 ± 0.52 g) or pollen substitute (5.68 ± 0.28 g), whereas 4.73 ± 0.13 g in sugar syrup feeding colonies (**Fig 5A**).

The article "Evaluation of queen cell acceptance and royal jelly production between hygienic and non-hygienic honey bee (Apis mellifera) colonies" was retracted in 2022. Reasons: compromised peer review; a conflict of interest; concerns about the authorship.

**Fig 5:** The nutritional effect on royal jelly (shows as mean ± SE) production between hygienic and non-hygienic colonies. (a) RJ yield in grams/ colony after 72 h of harvesting, (b) RJ yield in mg/ cell cup between both bee stocks.

In addition, the nutritional effect on RJ yields per cell cup was investigated between hygienic and non-hygienic colonies (**Fig 5B**). In hygienic bee colonies, no significant difference is present in RJ production per cell cup those fed on either pollen diet or pollen substitute (**Fig 5B**). In hygienic beelines, the RJ yield was 239.62 ± 2.74 mg/cup cell, 235.89 ± 3.55 mg/cup, and 221.48 ± 2.55 mg/cup in the case of natural pollen diet, pollen substitute, and sugar syrup fed colonies, respectively. In non-hygienic bee stock, the maximum mean weight of RJ production was 160.39 ± 4.36 mg/cup in pollen diet, while 153.45 ± 3.16 mg in pollen substitute and less RJ yield was 141.54 ± 2.17 mg/cup in sugar syrup feeding colonies (**Fig 5B**).

## Discussion

This study is performed to identify the larval acceptance rate and mean weight of RJ production between hygienic and non-hygienic lines. Our results demonstrated that mean percentage of larval acceptance rate and mean weight of RJ yield was statistically greater in hygienic lines as compared to non-hygienic bee colonies. Past studies reported that production of bee product such as pollen and RJ does not seem to be incompatible with hygienic behavior [46, 47].

Our findings showed that the queen cell acceptance rate was 64.33 ± 2.91% in the hygienic bee stocks and 29.67 ± 1.20% in non-hygienic bee stocks. The RJ yield was 12.23 ± 0.52 g and 6.72 ± 0.33 g in hygienic and non-hygienic colonies, respectively. In addition, the highest RJ yield was 234. 99 ± 2.22 mg/cell cup in hygienic bee colonies and, whereas 158.87 ± 2.52 mg/ cell cup in non-hygienic bee colonies. Previous literature indicated a lot of variations in RJ production, larval acceptance, and quality which affected my multiple factors including genetic variations, harvesting time, queen fecundity, and other environmental factor associated to weather condition and feeding conditions [21, 33, 38, 48–50]. For instance, a previous literature reported that Africanized honeybees have a lot of variation, which opens up the possibility of selecting these honeybees for any production, such as honey, wax, pollen, propolis, or RJ, as happened with European honeybees selected to pollinate alfalfa cultures in the United States [51, 52]. Another research investigated the larval acceptance and RJ yield between two races such as high royal jelly producing bees (RJBs) and Italian bees (ITBs), the mean RJ yield was 54.0 ± 3.4 g in RJBs while 3.7 ± 0.84 g in ITBs. The larval acceptance rate was (75%) was more in RJBs than ITBs that was (10%) [19]. These results are inconsistent with our findings, that showed that larval acceptance rate and RJ yield was low as compared to RJBs and more than ITBs. RJ production higher in RJBs suggested that honey bees’ lines effect on larval acceptance and RJ productions [19, 31]. Our results are in line with previous research, recorded that larval acceptance rate and per cell cup were 72.1% and 236.31 mg/cell cup for Italian bees and 65.43% and 187.24 mg/ cell cup in Carniolan bees [53]. Further, another study reported the mean larval acceptance rate and RJ yield was more in Carniolan than other races [41]. However, in our experiment, the RJ yield is lower than the other bees’ races that have been genetically engineered in other parts of regions worldwide.

The article "Evaluation of queen cell acceptance and royal jelly production between hygienic and non-hygienic honey bee (Apis mellifera) colonies" was retracted in 2022. Reasons: compromised peer review; a conflict of interest; concerns about the authorship.

Moreover, our result elucidates that the larval acceptance rate and RJ yield were significantly more in both bee stocks those fed on natural pollen diet. But larval acceptance rate and amount of RJ yield do not show statistically significant difference among both bee stocks those fed either natural pollen or pollen substitute diet. Therefore, artificial sugar supplementation during RJ yield is a typical beekeeping method, especially in regions where the temperature is particularly hot and dry. However, artificial supplementation of bees during RJ production is still a contentious topic. Surprisingly, our findings did not reveal the effect of different diets on the quality of RJ and their composition. Interestingly, for RJ quality, its major ingredients including water, protein, and 10-HDA remain constant between the bee colonies that fed pollen substitute when compared with control RJ samples [54]. For international market prospective, all major components of RJ are very important parameters of its quality to attract consumers. For example, if RJ has low content of 10-HDA, resulting reduce the consumers attraction and price of RJ in the market [28].

However, more research is required for better understand how different biotic and abiotic factors affect the larval acceptance and RJ yields in different bees’ races.

The article "Evaluation of queen cell acceptance and royal jelly production between hygienic and non-hygienic honey bee (Apis mellifera) colonies" was retracted in 2022. Reasons: compromised peer review; a conflict of interest; concerns about the authorship.

## Conclusions

Our result indicated that uncapped and removal percentage of dead broods was statistically more in hygienic lines as a comparison to non-hygienic bee colonies. Our results showed that larval acceptance rate, RJ yield per colony and per cell cup was significantly difference between both bee stocks. Moreover, the RJ yield per colony and per cell cup was not statistically significant between both bee stocks either fed on commercially available pollen or pollen substitute diet. In future, more research is required to unveil the quality and ingredients of RJ that gained from various diet source between hygienic and non-hygienic bee colonies.
